The article "Motor Imagination of Lower Limb Movements at Different Frequencies" was published in 2021. Journal: J Healthc Eng.

# Motor Imagination of Lower Limb Movements at Different Frequencies

**DOI:** 10.1155/2021/4073739

**Published:** 2021-12-22

**Authors:** Yingtao Liu, Chao Chen, Abdelkader Nasreddine Belkacem, Zhiyong Wang, Longlong Cheng, Chun Wang, Yuexiao Chang, Penghai Li

**Affiliations:** ^1^School of Integrated Circuit Science and Engineering, Tianjin University of Technology, Tianjin 300384, China; ^2^Key Laboratory of Complex System Control Theory and Application, Tianjin University of Technology, Tianjin 300384, China; ^3^Department of Computer and Network Engineering, College of Information Technology, UAE University, Al Ain 15551, UAE; ^4^China Electronics Cloud Brain (Tianjin) Technology Co. Ltd., Tianjin 300309, China; ^5^College of Mechanical and Electrical Engineering, Beijing University of Chemical Technology, Beijing 100029, China

## Abstract

Motor imagination (MI) is the mental process of only imagining an action without an actual movement. Research on MI has made significant progress in feature information detection and machine learning decoding algorithms, but there are still problems, such as a low overall recognition rate and large differences in individual execution effects, which make the development of MI run into a bottleneck. Aiming at solving this bottleneck problem, the current study optimized the quality of the MI original signal by “enhancing the difficulty of imagination tasks,” conducted the qualitative and quantitative analyses of EEG rhythm characteristics, and used quantitative indicators, such as ERD mean value and recognition rate. Research on the comparative analysis of the lower limb MI of different tasks, namely, high-frequency motor imagination (HFMI) and low-frequency motor imagination (LFMI), was conducted. The results validate the following: the average ERD of HFMI (−1.827) is less than that of LFMI (−1.3487) in the alpha band, so did (−3.4756 < −2.2891) in the beta band. In the alpha and beta characteristic frequency bands, the average ERD of HFMI is smaller than that of LFMI, and the ERD values of the two are significantly different (*p*=0.0074 < 0.01; *r* = 0.945). The ERD intensity STD values of HFMI are less than those of LFMI. which suggests that the ERD intensity individual difference among the subjects is smaller in the HFMI mode than in the LFMI mode. The average recognition rate of HFMI is higher than that of LFMI (87.84% > 76.46%), and the recognition rate of the two modes is significantly different (*p*=0.0034 < 0.01; *r* = 0.429). In summary, this research optimizes the quality of MI brain signal sources by enhancing the difficulty of imagination tasks, achieving the purpose of improving the overall recognition rate of the lower limb MI of the participants and reducing the differences of individual execution effects and signal quality among the subjects.

The article "Motor Imagination of Lower Limb Movements at Different Frequencies" was published in 2021. Journal: J Healthc Eng.

## 1. Introduction

Recently, the method of simulating exercise has received extensive attention from the brain science and neuroscience fields. At the same time, a mode similar to simulated exercise is a kind of self-movement in the brain, that is, motor imagination [1–3]. Motor imagination (MI) is defined as having no movement of oneself, simply relying on one's own brain to perform the movement of imagining oneself [4]. In the process of MI, it can enhance the ability to activate a specific motor function area in the brain and then achieve the purpose of improving the motor function [5, 6]. In addition, motor imagination and actual action execution have similar cognitive processes, which can reveal the inner relationship between the neural mechanism of motor imagination and actual action execution [7]. MI has the characteristics of independence and spontaneity that do not depend on external stimuli and has been widely used in the neurorehabilitation of stroke patients, sports training, brain-computer interface, and other fields and has become a research hotspot [8].

By improving the patients' lower limb MI ability to facilitate the recovery of their leg motor function and increasing the leg rehabilitation training effect, MI has the potential to help home-based remote neurorehabilitation training for stroke patients under the technical support of 5G telecommunications. Since it is very important to quantify the value of ERD and may provide the basis and convenient way for evaluating the therapeutic effect of leg rehabilitation and motor skill training under the technical support of data intelligence. Home-based remote neurorehabilitation training and the status or recovery effect evaluating can reduce treatment costs and avoid preventable diseases especially during the outbreak of COVID-19.

Previous studies on MI have been focused on classifying the types of imagery associated with different body parts and converting them to the control of a prosthetic executor, for example, computer cursor, and have made significant progress in feature information detection and machine learning decoding algorithms [9, 10]. Nonetheless, a low overall recognition rate, large differences in individual execution effects, and variances in signal quality are still problems that must be solved, which impeded the application in home-based remote neurorehabilitation [8]. Studies by scholars have confirmed that high-frequency upper limb MI can enhance the intensity of MI by enhancing the difficulty of imagination tasks [11–14]; it could be also an effective way for lower limb MI and has potential value for leg motor rehabilitation and motor skill training [11–15]. However, given that the EEG signals of lower limb MI are difficult to identify, there are few reports on the study of lower limb MI with divergent frequencies [16, 17]. This study aims to investigate various frequency leg-raising imagination tasks for MI to compare high- and low-frequency lower limb MI and to ensure whether HFMI can increase the difficulty of imagination tasks, strengthen the activation ability of the brain motor neural network of the participants, and improve the MI implementation effect. The results suggest that HFMI can optimize the quality of the brain signal of MI, improve the recognition rate, and reduce the difference in individuals in some respects that may be beneficial to leg motor rehabilitation and motor skill training.

The article "Motor Imagination of Lower Limb Movements at Different Frequencies" was published in 2021. Journal: J Healthc Eng.

Section 2 deals with the methods and materials for building the proposed paradigm of the study. This experimental paradigm is based on noninvasive measurements.  Section 3 presents the results of the comparative analysis of the lower limb MI of HFMI and LFMI.  Section 4 discusses the differences between distinct tasks. Subsequently, the conclusion and the arrangement of future works are tackled.

## 2. Methods and Materials

### 2.1. Comparison Experiment

This paper mainly discusses the distinction in the EEG signals of the right leg motor imagination with different difficulties instructed by videos showing high- and low-frequency leg lifting and designs experimental schemes on the basis of the two forms of task guiding (Figure 1).

Figure 2 displays the experimental process. Before the start of the experiment, there is 5 second preparation, which corresponds to the ready phase of the experiment flowchart. The subjects needed to relax and rest for a short time and adjust their state to prepare for the experiment. They were also requested to watch and imagine the leg movements when the video of lifting the right leg started. In addition, they were required to imagine strictly with video actions on the process of MI in the first-person perspective. Before the MI, there will be a red circle on the screen to indicate that it will last for 1 second, and then the subjects will start the MI task induced by the video.

In the experiment, low-frequency MI and high-frequency MI appear randomly but appeared with the same probability, each accounting for 50% in order to ensure the participants took part in the MI test without any training disturbing influence.

The video displayed the right leg raising of the participants in a real scene video. When the video showed the right leg raising twice in 4 seconds (as shown in Figure 1(b)), the subjects performed LFMI. When the video displayed the right leg raising four times in 4 seconds (as shown in Figure 1(c)), the subject performed HFMI. The video of the right leg raising started from 1 second each time; the duration was 4 seconds; the screen exhibited a relax prompt of 4 seconds; and the experiment ended. The use of induced video actions was mainly to guarantee that all the subjects can perform the MI task strictly in the same mode, amplitude, and speed by following the same video in the test. Subjects had an obligation to imagine strictly with video action on the process of MI in the first-person perspective.

The article "Motor Imagination of Lower Limb Movements at Different Frequencies" was published in 2021. Journal: J Healthc Eng.

### 2.2. EEG Data Acquisition and Processing Methods

The EEG signals were collected from 10 healthy subjects (6 males and 4 females, aged 20–26 years old) who had not participated in EEG experiments before. Throughout the experiment, they were asked to put on an electrode cap, sit relaxed in chairs with armrests, and conduct HFMI and LFMI experiments as required. The experimental equipment SynAmps2 is an electrophysiological amplifier developed by Neuroscan Company. It has 64 channels, and the electrodeposition is set on the basis of the international 10/20 system. In the present study, the grounding electrode was placed in the central area of the head; the reference electrode was set at the tip of the nose; the sampling frequency was 1,000 Hz; and the band-pass filter was 0.1–200 Hz. The frequency band of the filter in the software of the acquisition device is between 0.1 and 200 Hz. We will pass the data saved offline through MATLAB and then perform band-pass filtering [18]. The filtering range is between 0.1 and 30 Hz. Before the experiment, it was ensured that the impedance of each electrode was under 5 k. The software scan 4.5 was also employed for high-quality data acquisition [19, 20].

Event-related desynchronization (ERD) enables the quantitative analysis of the brain electrical signals of motor imagination. The ERD phenomenon is the reduction of EEG energy in certain characteristic frequency bands of EEG signals. ERD quantitative analysis on EEG signals helps judge the intensity of motor imagination on the basis of the mean value of ERD [19]. The smaller mean value of ERD corresponds to the greater intensity of MI. To study the MI EEG in the characteristic frequency band, the average ERD value is calculated using the following formula:

(1) $$\begin{array}{c} \text{ERSP}\left(f,t\right)=\frac{1}{n}\sum_{k=1}^{n}\left(F_{k\;}{\left(f,t\right)}^{2}\right), \end{array}$$

where *n* is the number of experiments and *F*_*k* _(*f*, *t*) represents the *k*-th energy spectrum estimation at frequency *f* and time *t*. The current study mainly analyzed the ERSP value of related leads within 0–4 seconds and 1–30 Hz.

(2) $$\begin{array}{c} \text{ERD}=\;\frac{1}{N}\sum_{f=f_{1}}^{f_{2}}\sum_{t=t_{1}}^{t_{2}}\left(\text{ERSP}\left(f,t\right)\right). \end{array}$$

This study employed the frequency-domain energy spectrum to analyze the EEG signals to describe the EEG signals thoroughly from the perspective of the frequency domain. This method is suitable for measuring nonlinear and complex signals and, thus, can accommodate the analysis of dynamic EEG signals. The frequency-domain energy spectrum can clearly show the energy change of the EEG signal, and its basic principles are as follows.

The article "Motor Imagination of Lower Limb Movements at Different Frequencies" was published in 2021. Journal: J Healthc Eng.

For nonlinear EEG signals, a random variable *X* can be assumed to express its characteristics. The value of *X* should be set to {*x*_1_, *x*_2_,…, *x*_*n*_} (*n* > 1), and the corresponding probability *P* is expressed as follows:

(3) $$\begin{array}{c} P=\left\{p_{1},p_{2},\ldots ,p_{n}\right\},\;\left(0\leq p_{i}\leq 1\right)\left(i=1,2,\ldots ,n\right). \end{array}$$

The formula satisfies ∑_*i*=1_^*n*^*p*_*i*_=1, and *p*_*i*_ is the probability of the *i*-th time. With this probability feature formula, the average value of the nonlinear system state number can be expressed as follows:

(4) $$\begin{array}{c} H=-\sum_{i=1}^{n}p_{i}\ln\left(p_{i}\right). \end{array}$$

In this study, we replaced the probability in the time domain by the energy spectrum density in the frequency domain to obtain the expression of the energy spectrum in the frequency domain as follows [17, 21]:

(5) $$\begin{array}{c} H_{pse}=-\int \hat{p}\ln\left(\hat{p}\right)\text{d}\hat{p}, \end{array}$$

where $\hat{p}$ represents the frequency-domain energy spectrum density, which is based on the short-time Fourier transform and evolves through formula reasoning. It can describe the EEG signal, and the expression is as follows:

(6) $$\begin{array}{c} \hat{p}=\frac{{\left|{\text{STFT}}_{x}\left(\omega ,t\right)\right|}^{2}}{2\Pi }. \end{array}$$

From formula (6), the frequency-domain energy graph of the motor-imaging EEG signal can be achieved, and the characteristic frequency and its band can be obtained in the frequency-domain energy graph.

## 3. Data Analysis and Results

The present study uses the above methods to analyze the EEG data of the HFMI and LFMI of 10 subjects (*S*1–*S*10) according to time-frequency diagram analysis, frequency-domain energy analysis, ERD quantification, and CSP feature extraction. Studies have verified that lower limb HFMI activates the brain to a greater extent and obtains higher recognition rates than LFMI. This suggests that HFMI can better optimize the quality of the brain telecom source of MI.

The article "Motor Imagination of Lower Limb Movements at Different Frequencies" was published in 2021. Journal: J Healthc Eng.

### 3.1. Time-Frequency Diagram Analysis and Results of ERD

With the use of the time-frequency diagram method to analyze the EEG data of all the subjects, the ERD phenomena of HFMI and LFMI can be obtained, as shown in Figures 3(a) and 3(b), which, respectively, correspond to the HFMI and LFMI average time-frequency of the 10 subjects. Each average time-frequency graph is acquired by averaging the energy values of the 10 subjects. The ERD phenomena in the alpha and beta bands are marked between the red dashed lines and the black dashed lines, respectively.

Figure 3 confirms that the ERD phenomenon of HFMI in the alpha frequency bands (8–13 Hz) during 0–4 seconds is more evident than that of LFMI. The qualitative analysis of two-dimensional time-frequency atlas reveals that the ERD phenomenon caused by HFMI is more significant than that caused by LFMI. To further compare the rhythm characteristics of the ERD phenomenon caused by HFMI and LFMI, the frequency domain analysis of its EEG is then conducted.

### 3.2. Frequency-Domain Energy Analysis and Results

To further explore the ERD phenomenon caused by HFMI and LFMI in the alpha and beta bands, MATLAB programming is utilized to obtain the brain electrical energy and frequency-domain energy change curve according to formulas (1) and (6). The frequency corresponding to the minimum energy value in the figure is the characteristic frequency.  Figure 4 gives the average frequency-domain energy curves of the HFMI and LFMI of the 10 subjects.

The abscissa represents the frequency (Hz), and the ordinate represents the average value (dB) of the brain electrical energy of the 10 subjects in the corresponding frequency band within the zero to 4 second time period. The blue and green curves represent the change in the EEG energy of HFMI and LFMI with frequency; the purple and green curves represent the change in the EEG energy of HFMI and LFMI with frequency; the black horizontal dotted line represents the baseline; the purple dense vertical dotted line represents the characteristic frequency of HFMI; and the purple sparse vertical dotted line represents the characteristic frequency of LFMI.  Figure 4 shows the average frequency-domain energy curve of the HFMI and LFMI of the 10 subjects. The alpha frequency band of the HFMI-induced ERD phenomenon is wider than that of LFMI, and the HFMI drop rate is greater. The beta frequency band of HFMI triggering the ERD phenomenon is also wider than that of LFMI, and the HFMI has a greater decline rate.

### 3.3. Quantitative Analysis of EEG Rhythm Features and Results

With the use of the frequency-domain energy analysis method to analyze the EEG data of all the subjects, the alpha characteristic frequency of HFMI and LFMI for each subject can be obtained by their frequency-domain energy curves. The characteristic frequency is the frequency corresponding to the minimum energy value in frequency-domain energy curves. So Table 1 was obtained; the characteristic frequency bands and overlapping areas of the frequency in HFMI and LFMI can be statistically analyzed.

The article "Motor Imagination of Lower Limb Movements at Different Frequencies" was published in 2021. Journal: J Healthc Eng.

Table 1 shows the alpha and the beta characteristic frequencies of HFMI and LFMI for the 10 subjects *S*1–*S*10.

The average characteristic frequencies of HFMI and LFMI in the alpha band are 9 Hz and 10 Hz, respectively. The average characteristic frequencies of HFMI and LFMI in the beta frequency band are 18 Hz and 20 Hz, respectively.

In addition, as shown in Figure 5, the correlation analysis of the characteristic frequencies of HFMI and LFMI indicates that there is a significant correlation between the characteristic frequencies of HFMI and LFMI (*p*=0.0074 < 0.01; *r* = 0.945).

From Table 1, we can obtain the alpha and the beta characteristic frequency bands of the 10 subjects (*S*1–*S*10). After the quantitative analysis, the alpha characteristic frequency band of the HFMI of the 10 subjects is 8–13 Hz, and that of LFMI is 8–12 Hz; the beta characteristic frequency band of HFMI is 18–23 Hz, and that of LFMI is 17–21 Hz. The characteristic frequency band of HFMI is larger than that of LFMI. This shows that the EEG characteristics of HFMI are more significant than those of LFMI and that HFMI can optimize the quality of EEG sources better than LFMI.

Formulas (1) and (2) can be used to obtain the average ERD of the HFMI and LFMI of each subject on the alpha and beta characteristic frequency bands, and then statistical analysis gives the average of the data of the 10 subjects, the standard deviation (STD), and the *p*-value of paired *t*-tests and correlations [22].

Table 2 demonstrates the average ERD values of the alpha beta characteristic frequency bands. The first column in the table represents the sequence number of the subjects, and the second and third columns are the HFMI and LFMI of all the subjects in the alpha characteristic frequency band, respectively. The fourth and fifth columns are the average ERD values of the HFMI and LFMI of all the subjects in the beta characteristic frequency band, respectively. Table 2 exhibits that the ERD mean value of the overall characteristic frequency band of all the subjects in the HFMI is smaller than that of LFMI (−1.827 < −1.3487 and −3.4756 < −2.2891), which shows that the ERD phenomenon of HFMI is more significant than that of LFMI. Additionally, the STD value of HFMI is greater than that of LFMI (0.4960 < 0.5279), which displays that the difference in the ERD phenomenon among the HFMI subjects is smaller than that among the LFMI subjects.

The article "Motor Imagination of Lower Limb Movements at Different Frequencies" was published in 2021. Journal: J Healthc Eng.

The STD value of HFMI in the beta frequency band is greater than that of LFMI (0.6460 < 0.6725). In the beta characteristic frequency band, the difference in ERD values among the HFMI task participants is small, and the difference in ERD values among the LFMI task participants is small.  Figure 6 shows the statistical analysis produced *p*-values and *r*-values of HFMI and LFMI in the alpha and beta frequency bands obtained by statistical analysis.  Figure 6(a) illustrates that the ERD mean values of HFMI and LFMI are significantly correlated with the alpha band (*p*=0.001 < 0.01; *r* = 0.811).  Figure 6(b) displays the correlation of the ERD mean between HFMI and LFMI in the beta frequency band (*p*=0.0002 < 0.01; *r* = 0.212). In addition, Figure 5 depicts that the characteristic frequencies of HFMI and LFMI are significantly correlated with a frequency range of 0–30 Hz (*p*=0.0074 < 0.01; *r* = 0.945).

### 3.4. Feature Extraction and Classification Analysis and Results

For the analysis of the recognition rate of the EEG signals induced by HFMI and LFMI more straightforwardly, the 8–30 Hz band EEG signals with the significant ERD phenomenon are selected in this study.

The researcher intercepts the attention signal segment evoked by motor imagination corresponding to the EEG signal and conducts an offline evaluation of its recognition rate. The common spatial pattern (CSP) was used for feature extraction and support vector machine (SVM) was used for classification [23–25].

CSP is a technique for extracting characteristic signals from multilead data under different types of conditions. It has a good filtering effect on the characteristics of motor imaging EEG signals [23, 24]. We diagonalize the covariance matrices of the two types of EEG signals at the same time and use the principal component analysis method to select different parts of the two types of covariance matrices and remove the overlapping parts to highlight the state. After the two types of original signals are filtered, a new timing distribution was generated. At the same time, this enhances the difference between the two types of EEG signals and suppresses noise. The formula of the filtered EEG signal *X*_CSP_ is expressed as follows:

(7) $$\begin{array}{c} X_{\text{CSP}}=W^{T}*X, \end{array}$$

where *X* is the original EEG signal, *W* is the matrix filtered by CSP, and *W* satisfies.

The SVM was used to calculate the recognition rate of motor imagination [26]. For the SVM-based classification, the “rbf” kernel function was set with a *C* value as (0.001, 0.01, 0.1, 1); gamma = “auto”; grid research was performed; and the best parameter *C* was selected through training to determine the optimal classification hyperplane. By considering the grid search algorithm, the classification was implemented with a tenfold stratified cross-validation. Finally, the prediction on the testing set of the classification model in each fold with optimal hyperparameters was evaluated [27, 28].

The article "Motor Imagination of Lower Limb Movements at Different Frequencies" was published in 2021. Journal: J Healthc Eng.

The SVM is employed to calculate the recognition rate of the two task modes, namely, HFMI and LFMI as follows [26–29]:

(8) $$\begin{array}{c} f\left(x\right)=\text{sgn}\left(\omega *x+b\right)=\text{sgn}\left(\sum_{i=1}^{l}a_{i}y_{i}\left(x_{i}*x\right)+b\right). \end{array}$$

The derived filter is adopted to obtain the characteristic value of the training sample and the test samples, which are all EEG signals selected from 1–4 second HFMI and LFMI. Then the characteristic value of the test sample is used for classification and recognition, and finally, the recognition rate is produced (as shown in Table 3). Table 3 represents 10 subjects and their recognition rate, mean, and STD of HFMI and LFMI. The average recognition rates of HFMI have reached 87.84%, and that of LFMI has reached 76.46%, which have exceeded the globally recognized available level (70%). The STD of recognition rates in HFMI is 0.00318, less than that of LFMI (0.00669), which suggests that individual difference of recognition rates among the subjects is smaller in the HFMI mode than in the LFMI mode.

In addition, statistics on the recognition rates of HFMI and LFMI (as shown in Figure 7) show that the recognition rates of HFMI and LFMI are significantly different (*p*=0.0034 < 0.01; *r* = 0.429).

## 4. Discussion and Conclusion

In the current study, the experimental paradigms of HFMI and LFMI are compared, and the research results confirm that the rhythm characteristics of HFMI EEG are more significant than those of LFMI. Among them, the ERD phenomenon of HFMI is more significant than that of LFMI. The frequency-domain energy curve of HFMI has a larger decline than that of LFMI. HFMI and LFMI are separable, and the recognition rate of HFMI is higher than that of LFMI.

On the basis of the motion imagination induced by live-action videos, the difficulty of imagination tasks is distinguished by imagining various frequencies of leg-lifting movements. In the preparatory experiment, twice leg lifts in 4 seconds are set as a low-frequency leg lift, which is the lower limit frequency; four times lifts in 4 seconds are the high leg lift frequency, which is the upper limit frequency. This study is conducted by comparing the two experimental paradigms of HFMI and LFMI: the time-frequency diagram shows that from the beginning of the two types of the experimental tasks of HFMI and LFMI to the end of the task (*t* = 0–4 second), the ERD phenomenon induced by HFMI is more significant than that of LFMI (as shown in Figure 3). Because the ERD phenomenon can truly reflect the activity state of cerebral cortex neurons, the motor imagination task does not require the subjects to perform any exercises, and the subjects must inhibit their own motor behaviors and complete the motor imagination tasks at the same time. As the difficulty of imagination increases, the subjects exert greater inhibition activities to prevent the occurrence of the exercise behavior of performing the movement, resulting in a significant ERD phenomenon. The ERD phenomenon is that when a person performs imaginary limb movements, the EEG signal of the corresponding brain area is inhibited, which leads to an evident and short-term energy attenuation in a specific frequency band. The imagination task of HFMI is comparatively more difficult; hence, HFMI has a stronger activation state of cortical neurons in the sensory-motor area of the brain. Therefore, the motor imagination intensity of HFMI is greater than that of LFMI.

The article "Motor Imagination of Lower Limb Movements at Different Frequencies" was published in 2021. Journal: J Healthc Eng.

In addition, Table 2 affirms that the ERD mean value of all the subjects' overall characteristic frequency bands is smaller in HFMI than that in LFMI (−1.827 < −1.3487 and −3.4756 < −2.2891). From the frequency-domain energy curve, the ERD phenomenon can be analyzed very intuitively (as shown in Figure 4). The ERD phenomenon in the alpha and beta bands corresponds to the energy attenuation of the energy curve. The drop amplitude of the frequency-domain energy curve of HFMI is larger than that of the low-frequency leg lift energy curve, which shows that the HFMI energy attenuation is more significant than the LFMI energy attenuation. The alpha characteristic frequency band of HFMI is 8–13 Hz, and the alpha characteristic frequency band of LFMI is 8–12 Hz; the beta characteristic frequency band of HFMI is 18–23 Hz, and the beta characteristic frequency band of LFMI is 17–21 Hz. The characteristic frequency band of HFMI is larger than that of LFMI. The EEG rhythm characteristics of HFMI and LFMI can reflect the activation state of the brain sensorimotor neural network, which shows that HFMI activates the brain sensorimotor neural network state more significantly than LFMI and that HFMI can optimize the quality of brain telecommunication sources better than LFMI. In the alpha bands, the STD value of HFMI is smaller than that of LFMI (0.4960 < 0.5279), so does in beta bands (0.6460 < 0.6725), and the ERD intensity individual difference among the subjects is smaller in the HFMI mode than in the LFMI mode.

The article "Motor Imagination of Lower Limb Movements at Different Frequencies" was published in 2021. Journal: J Healthc Eng.

Our aim is mainly focused on the development of various frequency leg-raising imagination tasks for the improvement of MI signals, so we just use the conventional approach, CSP-SVM [27, 28]. Notably, we acknowledged the existence of numerous alternative novel algorithms for decoding neural features of the MI EEG signal, such as filter bank common spatial pattern (FBCSP), EEG channel optimization, EEG channel optimization, internal feature selection method of CSP, and deep learning [23, 24]. In addition, the average recognition rate of HFMI (87.02%) is higher than that of LFMI (76.14%), which suggests the better MI implementation effect was gotten in HFMI. The STD of recognition rates in HFMI (0.00318) is less than that of LFMI (0.00669), which suggests that individual difference of recognition rates among the subjects is smaller in the HFMI mode than in the LFMI mode.

In this article, the comparative study of high- and low-frequency leg-raising video-induced lower limb MI is presented; HFMI can increase the difficulty of imagination tasks and improve the MI effect. Therefore, the characteristic frequency band and rhythm characteristics of HFMI and LFMI are significantly different, and the ERD phenomenon of HFMI is more evident than that of LFMI. The recognition rate of HFMI is higher than that of LFMI. Our findings suggest an application to optimize the quality of MI brain telecommunication sources by enhancing the difficulty of imagination tasks, thereby achieving the purpose of improving the overall recognition rate of the participants' lower limb MI and reducing the individual differences, which have the potential to help home-based remote neurorehabilitation training for the functional recovery of stroke patients under the technical support of big data intelligence and telecommunications [6, 30, 31]. Movement kinematics has been shown in nonhuman primate studies of hand reaching or drawing tasks, the direction, speed, and other information, so various kinematic parameters of the leg movement MI such as strength and amplitude can be performed to enhance the difficulty of imagination tasks and efficient training for subjects in future works [14, 31–34].

## Figures and Tables

**Figure 1:** Participants' right leg raising at different frequencies: (a) stationary leg, (b) low frequency of leg lifting, and (c) high frequency of leg lifting.

**Figure 2:** Experimental flowchart.

**Figure 3:** ERD phenomenon of the time-frequency diagram: (a) HFMI's ERD diagram and (b) LFMI's ERD diagram.

**Figure 4:** Average frequency-domain energy curves of HFMI and LFMI.

The article "Motor Imagination of Lower Limb Movements at Different Frequencies" was published in 2021. Journal: J Healthc Eng.

**Figure 5:** Correlation analysis of characteristic frequency between the HFMI and LFMI of 10 subjects.

**Figure 6:** ERD mean value and correlation of HFMI and LFMI in alpha and beta frequency bands: (a) the ERD mean value and correlation of HFMI and LFMI and (b) the ERD mean value and correlation of HFMI and LFMI in the alpha band in the beta band.

**Figure 7:** Statistical analysis of the recognition rate of HFMI and LFMI of the 10 subjects.

**Table 1:** Characteristic frequencies of the alpha and beta bands of the HFMI and LFMI of the 10 subjects.

Participant	HFMI's alpha characteristic frequency (Hz)	LFMI's alpha characteristic frequency (Hz)	HFMI's beta characteristic frequency (Hz)	LFMI's beta characteristic frequency (Hz)
*S*1	9	10	19	19
*S*2	10	11	17	20
*S*3	8	9	19	21
*S*4	10	11	17	20
*S*5	10	11	18	21
*S*6	8	9	19	19
*S*7	10	10	17	20
*S*8	8	9	18	21
*S*9	9	10	19	19
*S*10	8	10	17	20
Mean	9	10	18	20

**Table 2:** Average ERD values of alpha and beta characteristic frequency bands.

Subject	Alpha		Beta	
	HFMI	LFMI	HFMI	LFMI
*S*1	−2.105	−1.1209	−3.2531	−2.3827
*S*2	−1.1536	−1.0336	−3.9198	−2.5407
*S*3	−1.8398	−1.015	−3.8286	−1.6239
*S*4	−2.4525	−1.5579	−3.5187	−2.4161
*S*5	−1.9261	−1.3741	−3.9149	−3.4839
*S*6	−2.8428	−2.7137	−3.865	−2.3341
*S*7	−1.7287	−1.4509	−3.5315	−2.0094
*S*8	−1.6163	−1.0637	−2.1449	−1.2393
*S*9	−1.5344	−1.2998	−2.303	−1.7632
*S*10	−1.4708	−0.8574	−4.2069	−3.0973
Mean	−1.827	−1.3487	−3.4756	−2.2891
STD	0.4960	0.5276	0.6460	0.6725
*p*	0.001		0.0002	

**Table 3:** Overall recognition rate, STD, and the mean of the two tasks.

Participant	The recognition rate of HFMI	The recognition rate of LFMI
*S*1	0.91	0.90
*S*2	0.82	0.74
*S*3	0.75	0.73
*S*4	0.94	0.74
*S*5	0.85	0.65
*S*6	0.94	0.88
*S*7	0.94	0.78
*S*8	0.88	0.63
*S*9	0.88	0.78
*S*10	0.90	0.83
Mean	0.8784	0.7646
STD	0.00318	0.00669

## Data Availability

The experiment data are not available online for further research but available on reasonable request according to the policy of Tianjin University of Technology.
